The article "3D craniofacial registration using thin-plate spline transform and cylindrical surface projection" was retracted in 2025. Reasons: concerns about the results or conclusions; concerns about the peer review; concerns about the article.

# 3D craniofacial registration using thin-plate spline transform and cylindrical surface projection

**DOI:** 10.1371/journal.pone.0185567

**Published:** 2017-10-05

**Authors:** Yucong Chen, Junli Zhao, Qingqiong Deng, Fuqing Duan

**Affiliations:** 1 College of Information Science and Technology, Beijing Normal University, Beijing, China; 2 School of Data Science and Software Engineering, Qingdao University, Qingdao, China; University College London, UNITED KINGDOM

## Abstract

Craniofacial registration is used to establish the point-to-point correspondence in a unified coordinate system among human craniofacial models. It is the foundation of craniofacial reconstruction and other craniofacial statistical analysis research. In this paper, a non-rigid 3D craniofacial registration method using thin-plate spline transform and cylindrical surface projection is proposed. First, the gradient descent optimization is utilized to improve a cylindrical surface fitting (CSF) for the reference craniofacial model. Second, the thin-plate spline transform (TPST) is applied to deform a target craniofacial model to the reference model. Finally, the cylindrical surface projection (CSP) is used to derive the point correspondence between the reference and deformed target models. To accelerate the procedure, the iterative closest point ICP algorithm is used to obtain a rough correspondence, which can provide a possible intersection area of the CSP. Finally, the inverse TPST is used to map the obtained corresponding points from the deformed target craniofacial model to the original model, and it can be realized directly by the correspondence between the original target model and the deformed target model. Three types of registration, namely, reflexive, involutive and transitive registration, are carried out to verify the effectiveness of the proposed craniofacial registration algorithm. Comparison with the methods in the literature shows that the proposed method is more accurate.

## Introduction

3D data registration [1,2] is a basic problem in computer vision, and it is widely used in 3D statistical shape analysis, shape matching and retrieval, and so on. Face registration is one of the very first issues in realms such as face recognition [3,4], craniofacial analysis [5,6], 3D face reconstruction [7,8] and other face related research [9,10]. Craniofacial registration is used to establish a point-to-point correspondence in a unified coordinate system among human face geometric models of different poses and sizes. One intuitive criterion qualifying a perfect registration is the correspondence correctness of facial anatomic landmarks such as the nose tip, eye corners, etc. However, the complexity of the face morphological changes makes the 3D craniofacial registration challenging.

The iterative closest point (ICP) algorithm [2] is one often-used approaches for 3D face registration [4,11,12]. It optimizes a rigid transform by iteratively searching the closest points between two 3D point sets. ICP usually falls into the local optimum due to its local iteration, and the initialization quality also critically affects its performance. Yang et al.[13] proposed a globally optimal solution to 3D data registration by combining ICP with branch-and-bound (BnB), a global searching scheme. Alyüz et al. [4] performed a regional ICP registration for expression resistant 3D face recognition. Other researchers [14,15] also give variants of ICP. Although this research improves the performance of the ICP algorithm, the rigid transform nature of ICP cannot be changed. Registration based on ICP cannot fully capture the non-rigid shape variation among different human faces or expressions. In addition, when the model resolution changes dramatically, i.e., the face models of different data resources, the registration results by ICP may have many to one correspondence. Some researchers [16,17] project the 3D faces into 2D parameter space by surface parameterizations and realize the 3D registration via 2D matching. Generally, surface parameterizations suffer from the initialization of boundary points and the problem of structural consistency.

Compared with rigid transforms, non-rigid transforms such as affine, spline or radial functions can well-represent the shape variations of 3D craniofacial surfaces. The Thin Plate Spline transform (TPST) [18] is a widely used non-rigid transform for 3D face registration. It decomposes the deformation between two subjects into affine and non-affine components. The famous TPS-RPM method proposed by Chui and Rangarajan [19] incorporates TPS into the framework of ICP for matching two point sets. They iteratively performed a soft-assign and deterministic annealing optimization to compute point correspondence and used a binary correspondence matrix to record point matching. This method is sensitive to initial alignment and is not fit for the dense registration of 3D craniofacial models because running TPS with the whole dense point sets as control points is impractical. Hutton et al. [20] manually chose 9 facial landmarks as the control points to compute the TPS deformation between two 3D face models. Guo et al.[21] automatically annotated seventeen facial landmarks as the control points via PCA-based feature recognition combining 3D-to-2D data transformation. Schneider et al.[22] and Hu et al.[23] automatically selected a group of feature points as the TPS control points based on a rough registration of 3D faces using ICP. To establish the dense point correspondence between two faces, all of these methods need to perform ICP after the TPS deformation of the reference face.

In this paper, a 3D craniofacial registration method combining thin-plate spline transform and cylindrical surface projection is proposed. It can improve the registration accuracy and address the resolution inconsistency between 3D faces due to the cylindrical surface projection, which is a major flaw in methods in the literature. This paper is organized as follows. Section 2 analyzes the problem of facial registration in mathematics and gives its mathematical definition. Section 3 introduces the proposed algorithm in detail. Section 4 shows the experimental results. Section 5 concludes the work.

## Aspects of craniofacial registration

If not speaking in an exaggerated manner, a human craniofacial geometrical shape is as complex as that of coastlines of the Earth. A feasible treatment in facial registration is to cut off trivial complexities residing on a human face by viewing it as a two-dimensional, simply connected smooth manifold. This treatment of a human face gives its geometric modeling much more regularities; therefore, this treatment is followed hereinafter.

Mathematically, given a pair of human craniofacial models (labeled R for reference and T for target) with their corresponding two-dimensional smooth manifolds $F_{\text{R}}$ and $F_{\text{T}}$, respectively, the task of facial registration is to find a (possibly partial) smooth homeomorphism ${\text{H}}_{\text{RT}}:F_{\text{R}}↛F_{\text{T}}$ that conforms to a collection of predefined constraints. Among these constraints, the most intuitive is the correspondence of facial features as mentioned above. This requires several pairs of corresponding points with respect to each facial feature, $\left({\text{p}}_{\text{R}}^{\text{i}},{\text{p}}_{\text{T}}^{\text{i}}\right)$, where ${\text{p}}_{\text{R}}^{\text{i}}\in F_{\text{R}}$, ${\text{p}}_{\text{T}}^{\text{i}}\in F_{\text{T}}$ and i is the index for each pair. A registration H_RT_ under this constraint is subject to ${\text{p}}_{\text{T}}^{\text{i}}={\text{H}}_{\text{RT}}\left({\text{p}}_{\text{R}}^{\text{i}}\right)$. However, this constraint does not consider deformation of faces such as squeezing or stretching when the facial expression changes.

Any facial deformation due to facial expressions can also be ideally viewed as a smooth homeomorphism. Suppose that the deformations from R to R′ and T to T′ are smooth homeomorphisms ${\text{C}}_{{\text{RR}}^{\prime }}:F_{\text{R}}\to F_{{\text{R}}^{\prime }}$ and ${\text{C}}_{{\text{TT}}^{\prime }}:F_{\text{T}}\to F_{{\text{T}}^{\prime }}$, respectively. A bijective map ${\text{H}}_{{\text{R}}^{\prime }{\text{T}}^{\prime }}^{\prime }:F_{{\text{R}}^{\prime }}↛F_{\text{T}}$ is defined such that ${\text{H}}_{{\text{R}}^{\prime }{\text{T}}^{\prime }}^{\prime }={\text{C}}_{\text{T}{\text{T}}^{\prime }}\circ {\text{H}}_{\text{RT}}\circ {\text{C}}_{\text{R}{\text{R}}^{\prime }}^{-1}$. It can be verified that ${\text{H}}_{{\text{R}}^{\prime }{\text{T}}^{\prime }}^{\prime }$ is also a registration between R′ and T′, with their feature point pairs selected as $\left({\text{C}}_{{\text{RR}}^{\prime }}\left(p_{R}^{i}\right),{\text{C}}_{{\text{TT}}^{\prime }}\left(p_{T}^{i}\right)\right)$. In this case, H_RT_ and ${\text{H}}_{{\text{R}}^{\prime }{\text{T}}^{\prime }}^{\prime }$ are assumed to be equivalent with respect to the operator P∘(⋅) ∘ Q^−1^, which is defined as an equivalence relation with P and Q being any homeomorphism. Therefore, the concept of a facial registration is now generalized from H_RT_ to its equivalence class [H_RT_]. An algorithm is said to be a registration algorithm for H_RT_ if it outputs H_RT_(p) for every input p. A registration algorithm for H_RT_ is said to be perfect if it is also a registration algorithm for any other registration in [H_RT_]. So, a perfect registration algorithm exists if and only if there is a Turing-computable function for all registrations in [H_RT_]. Whether such a computable function exists or not is beyond the scope of this paper. However, if such a perfect algorithm exists, say A(p;R,T), it must hold to the following properties:

- Reflexivity: ∀R, ∀p ∈ R, such that p=A(p;R,R).
- Symmetry: ∀R, T, ∃p ∈ R, ∃q ∈ T, such that q=A(p;R,T)⇔p=A(q,T,R).
- Transitivity: ∀R,T_1_, T_2_, ∀p ∈ R, such that $A\left(\text{p};\text{R},{\text{T}}_{1}\right)=A\left(A\left(\text{p};\text{R},{\text{T}}_{2}\right);{\text{T}}_{2},{\text{T}}_{1}\right)$.

Actually, rather than seeking a perfect registration algorithm for all possible smooth deformations, a quasi-perfect algorithm is proposed only for non-serious deformations. To verify the effectiveness of the quasi-perfect algorithm, three types of registrations are naturally born from the above properties:

- Reflexive registration: this type of registration treats the same face R as both the reference face and the target face and then computes the difference between p and A(p;R,R), which is called the reflexive error.
- Involutive registration: this type of registration does registration back and forth between two distinct faces R and T, and it then computes the difference between p and A(A(p;R,T);T,R), which is called the involutive error.
- Transitive registration: this type of registration chains the registrations among three faces, treating T_2_ as a medium face, and then, it computes the difference between $A\left(\text{p};\text{R},{\text{T}}_{1}\right)$ and $A\left(A\left(\text{p};\text{R},{\text{T}}_{2}\right);{\text{T}}_{2},{\text{T}}_{1}\right)$, which is called the transitive error.

## The craniofacial registration algorithm

In brief, our algorithm for craniofacial registration can be divided into the following four phases:

1. Finding a cylindrical surface that best fits the reference craniofacial model. We gradually rotate, shift and scale a cylindrical surface by gradient descent to achieve best fitting toward the reference model.
2. Deforming the target craniofacial model to the reference model. By choosing a collection of corresponding feature point pairs on the reference and target models as control points, TPS can be used to deform the target to the reference model with an arbitrary smoothing parameter.
3. Deriving point correspondence between the reference and the deformed target model using CSP. We make use of the fitted cylindrical surface to derive a correspondence between the reference and deformed target models, where a time-consuming phenomenon emerges until unwrapping and straightening are employed.
4. Restoring the corresponding points on the original target craniofacial model from the points on the deformed target model.

### Cylindrical surface fitting of the reference craniofacial model

Although finding an appropriate cylindrical surface that fits a given face model best is actually a subjective mathematical game rather than an objective canonical routine, a precise procedure is still used to determine that surface. A normal practice is to fix the coordinate system of the reference craniofacial model and directly determine the algebraic surface equation. However, this equation may be hard to derive and handle due to its complex algebraic form. Instead, by keeping the central axis of the cylindrical surface always coinciding with X-axis of the Cartesian coordinate frame, we gradually rotate and shift the frame rigidly and adjust the radius of cylindrical surface, to attain a best fitting surface.

Here, Tait-Bryan angles are used to depict frame rotation. The frame is rotated from x-y-z to X-Y-Z; then, a translation is applied to X-Y-Z. The coordinate transform between system x-y-z and X-Y-Z is

$$\left(\begin{array}{c} w_{1}\\ w_{2}\\ w_{3} \end{array}\right)=\left(\begin{array}{ccc} 1 & 0 & 0\\ 0 & c_{3} & s_{3}\\ 0 & -s_{3} & c_{3} \end{array}\right)\left(\begin{array}{ccc} c_{2} & 0 & -s_{2}\\ 0 & 1 & 0\\ s_{2} & 0 & c_{2} \end{array}\right)$$

$$\left(\begin{array}{ccc} c_{1} & s_{1} & 0\\ -s_{1} & c_{1} & 0\\ 0 & 0 & 1 \end{array}\right)\left(\begin{array}{c} v_{1}\\ v_{2}\\ v_{3} \end{array}\right)-\left(\begin{array}{c} d_{1}\\ d_{2}\\ d_{3} \end{array}\right),$$ (1)

where (*v*_1_, *v*_2_, *v*_3_)^T^ are the coordinates in x-y-z, (*w*_1_, *w*_2_, *w*_3_)^T^ are the transformed coordinates in X-Y-Z, (*d*_1_, *d*_2_, *d*_3_)^T^ are the translation applied to X-Y-Z, *c*_1_ = cos *ψ*, *s*_1_ = sin *ψ*, *c*_2_ = cos *θ*, *s*_2_ = sin *θ*, *c*_3_ = cos *ϕ*, *s*_3_ = sin *ϕ*, and *ϕ*, *ψ*, *θ* are the angles rotated around the X, Y, Z-axis, respectively.

Define the deviation of a point from the cylindrical surface of radius *r* as ${\hat{\epsilon }}^{4}={\left(w_{1}^{2}+w_{2}^{2}-r^{2}\right)}^{2}$; then, the total deviation of the point cloud of the reference craniofacial model from that cylindrical surface with a system of constraints is (after some mathematical reductions) as follows:

$$\text{arg}\underset{r,\psi ,\phi ,d_{1},d_{2}}{\text{min}}\left\{\frac{1}{N}\overset{N}{\underset{i=1}{\sum }}\left({\hat{\epsilon }}_{i}^{4}\right)\right\},\;\text{s}.\text{t}.$$

$$\{\begin{array}{c} {\hat{\epsilon }}_{i}^{4}={\left(w_{i1}^{2}+w_{i2}^{2}-r^{2}\right)}^{2}\\ \left(\begin{array}{c} w_{i1}\\ w_{i2} \end{array}\right)=\left(\begin{array}{ccc} -s_{3} & c_{3} & 0\\ c_{3}s_{1} & s_{3}s_{1} & c_{1} \end{array}\right)\left(\begin{array}{c} v_{i1}\\ v_{i2}\\ v_{i3} \end{array}\right)-\left(\begin{array}{c} d_{1}\\ d_{2} \end{array}\right) \end{array}$$ (2)

where the subscript *i* indicates the *i*-th point.

Eq (2) is a mathematical optimization problem with five free variables, *r*, *ψ*, *ϕ*, *d*_1_, and *d*_2_. The analytic solution to Eq (2) is difficult to calculate. The numerical approach, i.e., gradient descent, is used to iteratively decrease the total deviation to its minima. Although *θ* (an angle rotated about the Z-axis) and *d*_3_ (the translation along the Z-axis) have no influence on this optimization problem, their values are chosen such that the centroid of the reference model is located on the XY-plane and the face direction is along the X-axis. This numerical iterative approach results in a perfect cylindrical surface fitting, as shown later in the experimental results.

### Craniofacial deformation using TPS

TPS is a flexible spline mapping function that has some desirable properties; the function is globally smooth and easy to compute. It has been widely used in data registration for various applications. For 3D face deformation, the TPS transformation can be defined as a smooth mapping *f* from R^3^ to R^3^. By choosing a set of corresponding landmark points {*L*_*Ri*_, *L*_*Ti*_}, i = 1,2,…,m on the reference and target faces as the controlling points, TPS minimizes the following bending energy function *E*(*f*) with the following interpolation conditions:

$$\begin{array}{l} E(f)={\int_{R^{3}}(\left(\frac{\partial^{2}f}{\partial x^{2}}\right)}^{2}+{\left(\frac{\partial^{2}f}{\partial y^{2}}\right)}^{2}+{\left(\frac{\partial^{2}f}{\partial z^{2}}\right)}^{2}+\\ 2{\left(\frac{\partial^{2}f}{\partial xy}\right)}^{2}+2{\left(\frac{\partial^{2}f}{\partial xz}\right)}^{2}+2{\left(\frac{\partial^{2}f}{\partial yz}\right)}^{2})dxdydz,\\ s.t.\;f\left(L_{Ti}\right)=L_{Ri},\;i=1,2,\ldots ,M \end{array}$$ (3)

TPS can be decomposed into affine and nonaffine components [24], i.e.,

f(P)=Pd+ϕ(P)Λ (4)

where P is the point on the target 3D face with homogeneous coordinate representation, d is a 4 × 4 homogeneous affine transformation matrix, **Λ** is a *M* × 4 non-affine warping coefficient matrix, and ϕ(P) = (ϕ_1_(P), ϕ_2_(P),…,ϕ_*M*_(P)) is a 1 × *M* kernel vector of TPS with the form ϕ_*k*_(P) = ‖P − *L*_*Tk*_‖.

If the interpolation conditions in Eq (3) are not strictly required, the following energy function can be minimized to find the optimal solution:

$$\bar{E}(\lambda \text{,}\Lambda ,\text{d})=\frac{1}{M}\sum_{j=1}^{M}\left\|f(L_{Tj})-L_{Rj}\right\|+\lambda E(f)$$ (5)

where λ is the smoothing regularization term. If λ is equal to zero, the interpolation conditions in Eq (3) are strictly satisfied. The TPS parameters d and **Λ** can be obtained by solving the following linear equation:

$$\left(\begin{array}{cc} \Phi & L_{R}\\ L_{R}^{T} & 0 \end{array}\right)\left(\begin{array}{c} \Lambda \\ d \end{array}\right)=\left(\begin{array}{c} L_{T}\\ 0 \end{array}\right)$$ (6)

Φ is a *M*×*M* matrix with the component Φ_*kl*_ = ‖*L*_*Tk*_ − *L*_*Tl*_‖, *L*_*R*_ is a *M*×*4* matrix with each row being the homogeneous coordinate of the point *L*_*Ri*_,*i* = 1,2,…,*M*, and *L*_*R*_ has the same meaning.

According to Eq (4), the target craniofacial model can be deformed to the reference model.

### Point correspondence deviation between the reference and target craniofacial models

Using TPST, the target craniofacial model is deformed and aligned to the reference model. Next, the point correspondence is established between the target and reference model via the cylindrical surface.

#### Straightforward derivation

Given a point Ω_*R*_ on the reference craniofacial model, the task of this phase is to determine a point $\bar{\Omega }$ on the deformed target craniofacial model that corresponds to Ω_*R*_. We make use of the fitted cylindrical surface *S*_*c*_ to determine $\bar{\Omega }$ by the intersection of some unknown triangular patch $\Delta \bar{A}\bar{B}\bar{\Gamma }$ of the deformed target craniofacial model and the projecting line $L_{\Omega_{R}}$ through Ω_*R*_ and some point of the same Z-coordinate on the central axis *PQ* of *S*_*c*_ (see Fig 1). Suppose that $L_{\Omega_{R}}$ intersects *S*_*c*_ at $\tilde{\Omega }\left({\tilde{\omega }}_{1},{\tilde{\omega }}_{2},{\tilde{\omega }}_{3}\right)$, which is called the CSP of Ω_*R*_; the task is to determine which triangular patch intersects $\;L_{\Omega_{R}}$. According to the projection mode, the coordinates of point $\bar{\Omega }$ should be $\left(k{\tilde{\omega }}_{1},k{\tilde{\omega }}_{2},{\tilde{\omega }}_{3}\right)$ with unknown *k*. It can be proved that $\Delta \bar{A}\bar{B}\bar{\Gamma }$ intersects $L_{\Omega_{R}}$ if and only if three coefficients $\bar{a}$, $\bar{b}$, and $\bar{c}$ as defined by Eq (7) are nonnegative, where the coordinates are $\bar{A}({\bar{\alpha }}_{1},\;{\bar{\alpha }}_{2},\;{\bar{\alpha }}_{3})$, $\bar{B}({\bar{\beta }}_{1},\;{\bar{\beta }}_{2},\;{\bar{\beta }}_{3})$, $\bar{\Gamma }({\bar{\gamma }}_{1},\;{\bar{\gamma }}_{2},\;{\bar{\gamma }}_{3})$, and $\tilde{\Omega }({\tilde{\omega }}_{1},\;{\tilde{\omega }}_{2},\;{\tilde{\omega }}_{3})$, respectively.

**Fig 1:** Correspondence between reference and TPST target craniofacial model.

$$\left(\begin{array}{c} \bar{a}\\ \bar{b}\\ \bar{c}\\ -\kappa \end{array}\right)={\left(\begin{array}{cccc} {\bar{\alpha }}_{1} & {\bar{\beta }}_{1} & {\bar{\gamma }}_{1} & {\tilde{\omega }}_{1}\\ {\bar{\alpha }}_{2} & {\bar{\beta }}_{2} & {\bar{\gamma }}_{2} & {\tilde{\omega }}_{2}\\ {\bar{\alpha }}_{3} & {\bar{\beta }}_{3} & {\bar{\gamma }}_{3} & 0\\ 1 & 1 & 1 & 0 \end{array}\right)}^{-1}\left(\begin{array}{c} 0\\ 0\\ {\tilde{\omega }}_{3}\\ 1 \end{array}\right)$$ (7)

Then, $\bar{\Omega }\left({\bar{\omega }}_{1},{\bar{\omega }}_{2},{\bar{\omega }}_{3}\right)$ is derived as a linear combination of $\bar{A}$, $\bar{B}$, and $\bar{\Gamma }$,

$$\left(\begin{array}{c} {\bar{\omega }}_{1}\\ {\bar{\omega }}_{2}\\ {\bar{\omega }}_{3} \end{array}\right)=\bar{a}\left(\begin{array}{c} {\bar{\alpha }}_{1}\\ {\bar{\alpha }}_{2}\\ {\bar{\alpha }}_{3} \end{array}\right)+\bar{b}\left(\begin{array}{c} {\bar{\beta }}_{1}\\ {\bar{\beta }}_{2}\\ {\bar{\beta }}_{3} \end{array}\right)+\bar{c}\left(\begin{array}{c} {\bar{\gamma }}_{1}\\ {\bar{\gamma }}_{2}\\ {\bar{\gamma }}_{3} \end{array}\right)=\left(\begin{array}{ccc} {\bar{\alpha }}_{1} & {\bar{\beta }}_{1} & {\bar{\gamma }}_{1}\\ {\bar{\alpha }}_{2} & {\bar{\beta }}_{2} & {\bar{\gamma }}_{2}\\ {\bar{\alpha }}_{3} & {\bar{\beta }}_{3} & {\bar{\gamma }}_{3} \end{array}\right)\left(\begin{array}{c} \bar{a}\\ \bar{b}\\ \bar{c} \end{array}\right),$$ (8)

or

$$\bar{\Omega }=\bar{a}\bar{A}+\bar{b}\bar{B}+\bar{c}\bar{\Gamma }.$$ (9)

The drawback of the straightforward derivation is that it is time consuming. For each point on the reference model, the intersection relationship between each triangular patch on the deformed target model and the projecting line of the point must be determined by Eq (7) to decide which patch intersects the projecting line of the point. Suppose there are *s* points on the reference model and *t* triangular patches on the target model; Eq (7) will be solved *s* × *t* times. This is a seriously intensive computation task when there are thousands of points on the reference model with thousands of small triangular patches of the target model, which characterize the straightforward derivation as time-consuming.

In fact, on one hand, the time-consuming phenomenon originates from the entanglement of $\;{\tilde{\omega }}_{l}$ with ${\bar{\alpha }}_{i},{\bar{\beta }}_{j},{\bar{\gamma }}_{k}$ in the same matrix, which is the first term on the right-hand side of Eq (7). If a method to disentangle ${\tilde{\omega }}_{l}$ from ${\bar{\alpha }}_{i},{\bar{\beta }}_{j},{\bar{\gamma }}_{k}$ can be found, this drawback can be excluded. Fortunately, disentanglement is found by unwrapping and straightening the 3D CSP image into a 2D planar image, which will lead to a good approximation of the straightforward derivation and make the correspondence derivation much more efficient. On the other hand, deciding the corresponding triangular patch in the deformed target model for each vertex on the reference model is more time-consuming. To streamline this procedure, we utilize the ICP algorithm to establish a rough point correspondence between the reference model and the deformed target model. Then, we consider only the K-neighborhood triangular patches of the corresponding point on the deformed target model for each vertex on the reference model. We set K as 2 in all experiments.

#### Unwrapping the CSP image and the straightening planar image

All points of the reference face and all small triangular patches of the deformed target face are projected onto the fitted cylindrical surface to obtain the projection image called the 3D *CSP image*. Then, the cylindrical surface as well as the CSP image are torn along a vertical generatrix without cutting any edge of small triangular patches. The image is unwrapped into a (2D) *planar image*. It is proven that the edges of the triangular patches of the deformed target face become planar arcs after unwrapping (see Fig 2).

**Fig 2:** Unwrapped planar image from the CSP image (yellow) and the straightened planar image (red).

Suppose that $\hat{\Omega }$ is the 2D point on the planar image originating from $\tilde{\Omega }$. It is obvious that $\Delta \bar{A}\bar{B}\bar{\Gamma }$ intersects $L_{\Omega_{R}}$ if and only if the planar arc-triangle $\hat{\Delta }\hat{A}\hat{B}\hat{\Gamma }$ contains $\hat{\Omega }$. Thus, the 3D geometrical problem of the straightforward derivation is transformed into an equivalent 2D planar geometrical problem. However, the irregularity and complexity of those arcs complicate the situation until it is proven that the arcs are not strictly curved due to the tininess of triangular patches of the deformed target face. Thus, we use straight line segments to approximate these arcs; all arcs are straightened by replacing them with straight-line segments (see Fig 2).

The straightened planar image can prove that $\Delta \hat{A}\hat{B}\hat{\Gamma }$ contains $\hat{\Omega }$, or equivalently $\Delta \bar{A}\bar{B}\bar{\Gamma }$ intersects $L_{\Omega_{R}}$, if and only if the three coefficients $\hat{a}$, $\hat{b}$, and $\hat{c}$ defined by Eq (10) are all nonnegative, where the coordinates are $\hat{A}\left({\hat{\alpha }}_{1},{\hat{\alpha }}_{2}\right)$, $\hat{B}\left({\hat{\beta }}_{1},{\hat{\beta }}_{2}\right)$, $\hat{\Gamma }\left({\hat{\gamma }}_{1},{\hat{\gamma }}_{2}\right)$, and $\hat{\Omega }\left({\hat{\omega }}_{1},{\hat{\omega }}_{2}\right)$, resepectively.

$$\left(\begin{array}{c} \hat{a}\\ \hat{b}\\ \hat{c} \end{array}\right)={\left(\begin{array}{ccc} {\hat{\alpha }}_{1} & {\hat{\beta }}_{1} & {\hat{\gamma }}_{1}\\ {\hat{\alpha }}_{2} & {\hat{\beta }}_{2} & {\hat{\gamma }}_{2}\\ 1 & 1 & 1 \end{array}\right)}^{-1}\left(\begin{array}{c} {\hat{\omega }}_{1}\\ {\hat{\omega }}_{2}\\ 1 \end{array}\right)$$ (10)

Similarly,$\;\hat{\Omega }$ is a linear combination of $\hat{A}$, $\hat{B}$, and $\hat{\Gamma }$,

$$\hat{\Omega }=\hat{a}\hat{A}+\hat{b}\hat{B}+\hat{c}\hat{\Gamma }.$$ (11)

Unlike Eqs (7) and (10) is much more efficient, because it successfully disentangles ${\hat{\omega }}_{l}$ from ${\hat{\alpha }}_{i},{\hat{\beta }}_{j},{\hat{\gamma }}_{k}$ by separating them into two matrices as the matrix and the vector on the right-hand side of Eq (10). This accelerates the coefficient computation greatly, since all points on the planar image originating from the reference face can be juxtaposed to right multiply that matrix as follows:

$$\left(\begin{array}{cccc} {\hat{a}}_{1} & \ldots & {\hat{a}}_{i} & \ldots \\ {\hat{b}}_{1} & \ldots & {\hat{b}}_{i} & \ldots \\ {\hat{c}}_{1} & \ldots & {\hat{c}}_{i} & \ldots \end{array}\right)\;={\left(\begin{array}{ccc} {\hat{\alpha }}_{1} & {\hat{\beta }}_{1} & {\hat{\gamma }}_{1}\\ {\hat{\alpha }}_{2} & {\hat{\beta }}_{2} & {\hat{\gamma }}_{2}\\ 1 & 1 & 1 \end{array}\right)}^{-1}\left(\begin{array}{cccc} {\hat{\omega }}_{11} & \ldots & {\hat{\omega }}_{1i} & \ldots \\ {\hat{\omega }}_{21} & \ldots & {\hat{\omega }}_{2i} & \ldots \\ 1 & \ldots & 1 & \ldots \end{array}\right),$$ (12)

where the subscript *i* indicates the *i*-th point. This juxtaposition allows for the coefficient computation for all points of the reference face toward a given triangular patch in only one matrix multiplication.

So far, Eq (11) only addresses the determination problem of the containing relationship or the equivalently intersecting relationship. However, the coordinates of the point $\bar{\Omega }$ or its coefficients $\bar{a},\bar{b},\bar{c}$ need to be determined. Using Eqs (7) and (8), the time-consuming phenomenon returns, however. Fortunately, for parallel projection, the following statement can easily be proven:

**Lemma 1.** *Coefficients* $\bar{a},\bar{b},\bar{c}$ are invariant under the parallel projections acting on $\bar{A},\bar{B},\bar{\Gamma }$, and $\bar{\Omega }$.

***Proof*.** Every parallel projection Prj can be viewed as a linear map P followed by a translation $\bar{\Delta }$, i.e.,$\forall x,\text{Prj}\left(x\right)=\bar{\Delta }+P\left(x\right)$. Also notice that $\bar{\Omega }=\bar{a}\bar{A}+\bar{b}\bar{B}+\bar{c}\bar{\Gamma }$ and $\bar{a}+\bar{b}+\bar{c}=1$.

Thus,

$$\begin{array}{l} \text{Prj}\left(\bar{\Omega }\right)=\bar{\Delta }+P\left(\bar{\Omega }\right)=\bar{\Delta }+P\left(\bar{a}\bar{A}+\bar{b}\bar{B}+\bar{c}\bar{\Gamma }\right)=\left(\bar{a}+\bar{b}+\bar{c}\right)\bar{\Delta }+\bar{a}P\left(\bar{A}\right)+\bar{b}P\left(\bar{B}\right)+\\ \bar{c}P\left(\bar{\Gamma }\right)=\bar{a}\left(\bar{\Delta }+P\left(\bar{A}\right)\right)+\bar{b}\left(\bar{\Delta }+P\left(\bar{B}\right)\right)+\bar{c}\left(\bar{\Delta }+P\left(\bar{\Gamma }\right)\right)=\bar{a}\text{Prj}\left(\bar{A}\right)+\bar{b}\text{Prj}\left(\bar{B}\right)+\bar{c}\text{Prj}\left(\bar{\Gamma }\right) \end{array}$$ (13)

The claim holds. ■

**Remark 1**. *The triangular patches of the deformed target face can be treated as the CSP as an approximate parallel projection because the patches are so small*. *This allows for the use of* $\hat{a},\hat{b},\hat{c}$ *to approximate* $\bar{a},\bar{b},\bar{c}$.

So, the following approximations may be used:

$$\bar{a}\approx \hat{a},\;\bar{b}\approx \hat{b},\;\bar{c}\approx \hat{c}.$$ (14)

Therefore,

$$\bar{\Omega }\approx \hat{a}\bar{A}+\hat{b}\bar{B}+\hat{c}\bar{\Gamma }.$$ (15)

Due to the juxtaposition (12) and approximations (14) (15), the unwrapping and straightening can result in a timesaving correspondence derivation.

#### Craniofacial registration

Since the objective of the TPS transform is to minimize the bending energy function between two surfaces, it is an invertible transform. When the point correspondence between the reference and the deformed target craniofacial models are established, the corresponding points to the target model can be restored using the inverse TPS transform determined by the initial control points in the reference and the target craniofacial models. In the matter of mathematics, an invertible transform keeps a linear combination of a set of vectors invariant. Assume $\hat{\Omega },\;\hat{A},\hat{B},\hat{\Gamma }$ and Ω, A, B, Γ are a group of corresponding points between the deformed target craniofacial model and the original target craniofacial model, i.e., $\hat{\text{X}}=\emptyset \left(\text{X}\right)$, and ∅ is the TPS transform. Thus, according to Eqs (11) or (15),

$$\Omega =\hat{\text{a}}\text{A}+\hat{\text{b}}\text{B}+\hat{\text{c}}\Gamma .$$ (16)

Finally, according to the point correspondence between the reference and target models, we can determine the rotation, translation and scale between them and obtain the point correspondence in a unified coordinate system.

## Experiments and discussions

The proposed method is validated with two datasets. The first dataset is BU-3DFE [25], which includes 3D face models of 25 different expressions of 100 subjects, including 56 males and 44 females, and each face model includes several thousand vertices plus 83 feature points. The other dataset is the craniofacial dataset used in [6] in which each craniofacial model has more than 40000 vertices. Our research was approved by the Institutional Review Board (IRB) of the Image Center for Brain Research, National Key Laboratory of Cognitive Neuroscience and Learning, Beijing Normal University. All participants provided informed written consent to publish the experimental images as outlined in the PLOS consent form.

### BU-3DFE

These data is used to verify the effectiveness of the proposed method. From the dataset, 4 female faces labeled F0005, F0020, F0023, F0029 and 4 male faces labeled M0009, M0011, M0042, M0043 are randomly selected to verify the effectiveness of the proposed algorithm. Registration is completed every round for a pair of faces, treating each as the reference face and the other as the target face, for a total of 56 rounds. Only one round between M0042 and M0043 is presented in this work, where M0042 is the reference face and M0043 is the target face.

First, CSF is applied to reference face M0042. The deviation and gradient norm are iteratively decreased by gradient descent (Fig 3). Because the cylindrical surface axis always coincides with the Z-axis during optimization, the fitted face finally postures upright in the new coordinate system. However, CSF is sensitive to the spatial distribution of the reference face points. This encourages the removal of non-facial points, so only facial points are retained and are distributed evenly to achieve a most reasonable CSF.

**Fig 3:** The variation of deviation (cost) and norm of gradient with iteration in CSF for M0042.

83 control points are correspondingly marked on M0042 and M0043 (Fig 4). Then, TPST is applied to M0043 with respect to these control points to align it with M0042. To achieve a smoother transform, a nonnegative smoothing parameter λ is introduced. When λ = 0, the control points of M0043 are exactly transformed to those of M0042. When λ becomes greater, the transformed control points deviate further from those of M0042, but the transformed face becomes smoother.

**Fig 4:** M0043 and M0042 with control points.

Fig 5 shows the planar image with a small portion of outliers, which leads to a small portion of unregistered points for M0042 (Fig 6). In each round between two distinct faces, the percentage of unregistered points is approximately 5% ~ 15%. The unregistered points occupy the margin of M0042.

**Fig 5:** Planar image and control points of M0043 (green) and M0042 (blue) unwrapped from the CSP image.

**Fig 6:** Unregistered points of M0042, a proportion of 6.68%.

The Reg(T, R, λ) notation is used to denote the registration between reference face R and target face T where the smoothing parameter is λ. Fig 7 shows the result of the registration between M0042 and M0043.

**Fig 7:** Reg(M0043, M0042, 0.1).

To verify the effectiveness of the proposed registration algorithm, the distances of corresponding points are computed upon three types of registrations, i.e., reflexive, involutive, and transitive registrations.

In reflexive registration, the difference between M0043 and Reg(M0043, M0043, 0.1) is verified by computing the Euclid distance as the reflexive error between every two corresponding points. The reflexive errors histogram shows that nearly all corresponding points coincide, where the mean reflexive error is on the order of magnitude of 10^−15^. The spatial distribution of these reflexive errors shows that they are consistently very small (Fig 8).

**Fig 8:** Distribution of the reflexive error. Magnitudes from small to large are colored blue to red.

Similarly, in involutive registration, the difference between M0042 and Reg(M0042, Reg(M0043, M0042, 0.1), 0.1) is verified by computing the Euclid distance as the involutive error between every two corresponding points. The involutive error histogram shows that their distribution is not as concentrated as that of reflexive errors. The mean involutive error is poorer at a much greater order of magnitude of 10^−4^. The spatial distribution of these involutive errors shows that large errors (colored in red) occupy areas near the ears, small errors (colored in blue) occupy the most areas of the front, and medium errors (colored in green) occupy areas between the other two areas (Fig 9). Notice that slightly medium errors occupy the nose bulge area.

**Fig 9:** Distribution of involutive errors.

Large errors occupy the areas near the ears because of the non-existence of control points in these areas, which as a consequence cause bad alignments with the reference face in these areas after TPST. To diminish these errors, control points are added. Medium errors occupy the nose area because of the abrupt nose slope from relatively flat cheeks, which causes bad correspondence between points on nose when CSP is applied. To diminish these errors, CSP is separately applied to the nose area.

In transitive registration, M0011 is chosen as the medium face; then, the difference between Reg(M0043, M0042, 0.1) and Reg(M0043, Reg(M0011, M0042, 0.1), 0.1) is verified by computing the Euclid distance as the transitive error between every two corresponding points. The histogram and spatial distribution of transitive errors are similar to those of involutive errors (Fig 10).

**Fig 10:** Distribution of transitive errors.

We have also tried dozens of different λ values, but all the registration results are overall similar to the case when λ = 0.1. Therefore, we assume that the value of λ, to some extent, has little impact upon our registration algorithm.

### Craniofacial dataset

The craniofacial data are used to compare the proposed method with the TPS algorithm. From the dataset, one model is randomly chosen as the reference model, while four models are chosen as the target models. The face part in craniofacial reconstruction is the primary focus, so the back part of the reference craniofacial model is removed, as shown in Fig 11. Thus, the reference craniofacial model has 40969 vertices. In performing the TPS and the proposed method, we manually choose nine landmarks including four eye corners, one nose tip, two nasal base points and two mouth corners as control points. The registration results are shown in Fig 12. The first column displays the results of the four target models, and the other two columns show the superimpositions of the reference mode and the registered target models by TPS and the proposed method. The distance increases from blue to red. To compare the results qualitatively, we compute the minimum, maximum and mean of the distance of the corresponding points, and the results are shown in Table 1. It can be seen that the proposed method is more accurate than TPS. The TPS method performs ICP after the TPS deformation of the reference face, and it finds one corresponding point in the original sampling point set of the target for each point in the reference craniofacial model. The proposed method performs resampling in the target model to establish the point correspondence, which improves the registration accuracy.

**Fig 11:** Reference craniofacial model.

**Fig 12:** The registration results.

**Table 1:** Distance of corresponding points.

Index	Distance	TPS	Proposed method
**1**	**Min**	3.62462E-006	7.82084E-007
	**Mean**	0.21187	0.16238
	**Max**	0.74487	0.72554
**2**	**Min**	3.0453E-006	3.90217E-006
	**Mean**	0.16437	0.12914
	**Max**	0.73544	0.59786
**3**	**Min**	3.26623E-005	3.41959E-007
	**Mean**	0.24170	0.19271
	**Max**	0.92224	0.95777
**4**	**Min**	1.19654E-005	4.71466E-006
	**Mean**	0.14822	0.12997
	**Max**	0.77607	0.61540

Once the reference model is fixed, the cylindrical surface fitting in the proposed method needs to be performed only once, which decreases computational complexity. Moreover, TPST and ICP are performed by both the TPS method and the proposed method. Thus, more computation in the proposed method is needed to determine the CSP projection point of the reference model vertex on the deformed target model, i.e., determining the relationship between the CSP projection point and the triangle mesh, which increases the time cost of the proposed method by three times over that of the TPS method. Fortunately, it is a matter of indifference to craniofacial registration, since many craniofacial applications do not need real-time operations.

## Conclusions

In this paper, a non-rigid 3D craniofacial registration method using thin-plate spline transform and cylindrical surface projection is proposed. Most parts of our algorithm are about geometrics. This deterministic geometrical approach loses some variability in the registered face model, but its effectiveness is strongly supported by the registration results in the experiments. However, some weaknesses in the proposed registration algorithm still exist including the following. First, CSF depends on the point cloud of the reference face model. A certain proportion must be used, so non-facial points may influence the fitted cylindrical surface. Second, manually marking control points on a face model is laborious and very subjective from one person to another. Third, the application of the same TPST parameterization to a whole target face ignores the local topological variations that need different configurations. Finally, CSP is somewhat vulnerable to bumpy surfaces on human faces, such as nose bulge areas. To overcome the above weaknesses, a finely crafted reference face is necessary with automatic markings for better coverage of control points, and decomposition of the model into parts to which TPST and CSP are separately applied is an area to be studied in future research.
